The article "Aloe monticola Reynolds: A refugee of the mountains − contributing towards its conservation through in vitro propagation" was published in 2023. Journal: Heliyon.

# *Aloe monticola* Reynolds: A refugee of the mountains − contributing towards its conservation through *in vitro* propagation

**DOI:** 10.1016/j.heliyon.2023.e22955

**Published:** 2023-12-03

**Authors:** Birhanu Debesay Berhe, Desta Berhe Sbhatu, T. Mohammad Munawar, Gebreselama Gebreyohannes

**Affiliations:** Department of Biological and Chemical Engineering, Mekelle Institute of Technology, Mekelle University, PO Box 1632, Mekelle, Ethiopia

**Keywords:** Acclimatization, *Aloe monticola*, Initiation, *In vitro* propagation, Offshoots, Rooting, Shooting

## Abstract

*In vitro* micropropagation study of *Aloe monticola* Reynolds was conducted using offshoots in Murashige and Skoog (MS) media enriched with plant growth regulators (PGRs). Initiation experiment, carried out by culturing sterilized explants in full-strength MS media enriched with 0.0–1.0 mg/L benzyl amino purine (BAP) alone and in combination with 0.10 mg/L indole-3-butyric acid (IBA), resulted in 89 − 100 % healthy and live (i.e., initiated) explants in 9–29 days. Regeneration study, conducted by culturing initiated explants in full-strength MS media supplemented with 0.0–3.0 mg/L BAP alone and in combination with 0.50 mg/L IBA, showed that treatments enriched with 1.0–3.0 mg/L BAP in combination with 0.50 mg/L IBA yielded better shooting responses than the rest of the treatments. The rooting responses of the shoots were also tested by culturing in half-strength MS media enriched with 0.0–4.0 mg/L NAA alone and in combination with 0.25 mg/L IBA. Better rooting responses were observed in treatments supplemented with 1.0–4.0 mg/L NAA in combination with 0.25 mg/L IBA with two exceptions. The responses of *A. monticola* plantlets to primary and secondary acclimatization in greenhouse, nursery shade, and direct sunlight in coco peat, composted soil, and manured soil were excellent – with survival percentages of 90–98 %. The findings of this empirical research are important for developing refined protocol of *in vitro* micropropagation of this ecologically important but endangered plant.

## 1 Introduction

Species of the genus *Aloe* (Aloaceae) are widely used medicinal plants. They are often thought to grow in hot and dry climates only. But they actually grow in variety of habitats and climates including deserts, grasslands, coastal areas, and alpine locations. Likewise, they thrive in all soil types including in rocky or gravelly soils, richer soils among grasses, cracks and crevasses in rocks, and sandy soils [1]. The genus includes about 450–600 species throughout the planet and 50 species are known and described in Ethiopia and Eritrea so far; 31 of which being endemic to Ethiopia [[1], [2], [3]]. *A. monticola* Reynolds is one of these accepted species originated from Ethiopia. The specific epithet ‘monticola’ denotes the habitat of the species where ‘monti’ refers to mountain and ‘cola’ refers to dweller [1].

The demand for *Aloe* species is increasing progressively in the medicinal and cosmetic industries. But efforts to increase production to meet the demands are absent [[4], [5], [6], [7]]. For example, natural stand in the wild is not enough to meet demands in Ethiopia; and in many cases it is depleting quite quickly [8]. This is because aloes regenerate poorly. Their vegetative propagation is slow while their sexual reproduction by seeds is ineffective due to male sterility and genetic unpredictability. The vegetative propagation by offshoots takes place only during raining seasons. Frequent droughts and erratic rainfall due to climate change is making this process ineffective [1]. Large-scale *in vitro* propagation can be regarded as the most viable approach to fulfill the commercial demands and provide plantlets for assisted regeneration [9,10].

In addition to the industrial demand, many aloe species are threatened due to many problems of environmental degradation and climate change. Hence, Ethiopian aloes are highly threatened due to destruction of their natural habitats, unsustainable use or over exploitation for various purposes, destruction of the plants in harvesting, and high degrees of endemism in small restricted areas [2,11,12]. Nearly all Ethiopian aloes are listed in the CITES (Convention on the International Trade in Endangered Species of Wild Fauna and Flora) Appendix II implying that plants in the wild stand cannot be used for commercial purposes. Yet, many of them are put in the IUCN (International Union for Conservation of Nature) Red List as near vulnerable (3 species), near threatened (four species), and endangered (eight species).

*Aloe monticola*, an ecologically and environmentally restricted plant, is one of the endangered species due to its low regeneration capacity, environmental degradation by encroachment to its fragile habitat by humans, absence of soil and water conservation measures targeting it, and frequent droughts and erratic rains due to climate change. In Tigrai, Ethiopia, its natural stands are very small and are limited to highlands and ecologically fragile mountains cliff and plateaus. The growth of *A. monticola* offshoots to maturity takes several years. And yet, chances are high that its offshoots are eaten by livestock. Therefore, artificial propagation through *in vitro* methods to assist the regeneration of such species is the best and efficient approach [13,14]. The present study was aimed to develop a suitable and reproducible protocol for *in vitro* propagation and *ex vitro* establishment of *A. monticola* using offshoots as explants. The findings will assist efforts of large-scale production for commercial needs and environmental rehabilitation purposes.

## 2 Materials and methods

### 2.1 Description of experimental site

The study was conducted in Tigrai Biotechnology Center Pvt. Ltd. Co. Lab, formerly known as Mekelle Plant Tissue Culture Laboratory. The facility is located in Mekelle, Tigrai, Ethiopia (alt.: 1979 masl; lat.: 13° 30″ 0′ N; long.: 39° 28″ 11′ E) about 200 km southeast of the historic city of Aksum. The mean annual temperature of Mekelle city ranges from 16 °C to 20 °C.

### 2.2 Collection, preparation, and sterilization of plant materials

Healthy offshoots of *A. monticola* were collected from wild stand at the east bank of Aiba, Emba Alaje district, South Tigrai, Ethiopia (12.882 N, 39.549 E; alt.: 2750 masl). Healthy and vigorous mother plants with miniature offshoots were identified and 198 offshoots were carefully collected from the bases of the mother plants with minimum damage and contamination. The offshoots were trimmed to 2–3 cm long explants with two leaves and cleaned and sterilized according to the procedures established in the works of Niguse et al. [15], Hailu et al. [16], and Olivera et al. [17]. Cleaning of the explants was carried out by: (a) washing them with running tap water for 30 min to remove soils and debris from their surfaces; (b) washing them with distilled water for 30 min; (c) immersing them in a solution of Tween-20 and soap and shaking for 5 min, and (d) washing them in distilled water for 10 min to remove traces of the detergents.

Likewise, sterilization of the explants was carried out by: (a) soaking them in flask containing an aqueous solution of 0.25 % kocide (active ingredient: cupper hydroxide), 0.25 % ridomil (active ingredient: metalaxyl-m), and 0.25 % bayleton (active ingredient: triadimefon 50 %) for 10 min while shaking; (b) rinsing them gently with distilled water three times to remove chemical residues; (c) soaking them in 5 % NaOCl solution for 10 min; (d) rinsing them with distilled water three times to remove traces of chemicals, and (e) sterilizing them under laminar airflow cabinet by soaking and shaking in fresh soap solution. The soap solution was composed of sterile distilled water, 2 drops of Tween-20, and 0.25 % w/v HgCl_2_ aqueous solution. Finally, the explants were rinsed three times with sterile distilled water to remove traces of HgCl_2_ and were kept in sealed, sterile flasks till they were cultured in initiation media [[15], [16], [17]].

### 2.3 Preparation of MS growth media

A 1 L unit of full-strength Murashige and Skoog [18] (MS) medium was prepared by mixing and dissolving many constituents in double distilled water. It included stock solutions of: (a) macronutrients (20 mL), (b) micronutrients (5 mL), (c) calcium chloride (10 mL), (d) FeSO_4_.7H_2_O-NaEDTA.2H_2_O (10 mL), (e) myo-inositol (1 mL), (f) amino acids (10 mL), (g) PGRs (required volumes), (h) table sugar as C-source (30 g/L), and (i) agar as gelling agent (5 g/L). The agar, soluble at the boiling point of pure water, had gel strength of 700–1100 g/cm^2^ (with 1.5 % solution at 20 °C), viscosity of 10–100 cps (with 1.5 % solution at 60 °C), setting point of 32–45 °C, and melting point of 85–95 °C. The pH of all MS media were adjusted to 5.8 by adding drops of 1 N NaOH and 1 N HCl as required. Subsequently, 60 mL MS medium was dispensed into sterile 300 mL, 15 cm high magenta culture bottles and autoclaved at a temperature of 121 °C with a pressure of 15 psi for 15 min. The bottles holding sterilized media were transferred to media storage room for five days before use [[15], [16], [17],^19^].

### 2.4 *In vitro* and ex vitro experiments

#### 2.4.1 Initiation experiment

Twenty two (22) treatments were prepared in triplicates in magenta culture bottles containing full-strength MS media. The treatments were supplemented with 0.0 (control), 0.10, 0.20, 0.30, 0.40, 0.50, 0.60, 0.70, 0.80, 0.90, and 1.00 mg/L BAP alone and in combination with 0.1 mg/L IBA. Three explants were cultured in each bottle. The culture bottles were labeled, capped, and placed randomly in growth room racks; and maintained at 25 ± 2 °C temperature and under 16/8 h (light/dark) photoperiod with 2000 to 2500 lux light intensity [17,19]. The initiation experiment was run for 30 days. Days to initiation, number of explants initiated, number of clean and live explants, and number of explants that produced new microshoots were recorded for each treatment.

#### 2.4.2 Regeneration experiment

Fourteen (14) treatments were prepared in triplicate in magenta culture bottles. The treatments contained full-strength MS media enriched with 0.00 (control), 0.50, 1.00, 1.50, 2.00, 2.50, and 3.00 mg/L BAP alone and in combination with 0.50 mg/L. Initiated explants and microshoots were trimmed and excised into 2–3 cm long explants with two leaves. Five explants were cultured in each magenta culture bottle. The culture bottles were randomly placed in growth racks with similar temperature and light conditions to that of initiation experiment [15,16]. The shooting experiment was run for 60 days. Data on days to shooting were collected since the seventh day of culturing. Data on number shoots per explant, length of shoots, and number leaves per shoot were recorded at the end of the 60 days of culturing.

#### 2.4.3 Rooting experiment

Eighteen (18) treatments were prepared in triplicate in magenta culture bottles. The treatments contained half-strength MS media enriched with 0.00 (control), 0.5, 1.00, 1.50, 2.00, 2.50, 3.00, 3.50 and 4.00 mg/L NAA alone and in combination with 0.25 mg/L IBA. Healthy and vigor shoots were collected from the regeneration experiment and were trimmed into 2–3.5 cm long, 2-leaved shoots. Six shoots were cultured in each magenta culture bottle. The culture bottles were randomly placed on growth room racks with similar temperature and light conditions specified for initiation [15,16,19]. The rooting experiment was run for 30 days. Data on days to rooting were collected since the seventh day of culturing. Data on number of roots per plantlet, length of roots, and number of leaves per plantlet were collected at the end of the 30 days.

#### 2.4.4 Acclimatization experiment

*Ex vitro* study included primary and secondary acclimatization experiments [19]. Whereas primary acclimatization study was conducted in greenhouse with coco peat as planting material, secondary acclimatization studies were conducted in nursery shade and direct sunlight with composted and manured soils as planting materials. Whereas the composition the manured soil was forest soil, sand, and manure at 1:1:1 ratio, the composition of the composted soil was forest soil, sand, and compost at 1:1:1 ratio. The planting materials were filled into polyethylene bags (length 15 cm; diameter 9 cm) and prepared for planting.

Plantlets (rooted shoots) were carefully removed from the magenta culture bottles and washed with lukewarm (40 °C) tap water to reduce contaminants and remove the gelling agent. For the primary acclimatization study, 331 plantlets were planted on coco peat in 48-holes Pro tray and put on greenhouse bench. The plantlets were covered with white plastic sheet to maintain 80 − 90 % RH (relative humidity) and 25 ± 2 °C temperature for one week. In the second week, the plantlets were exposed to greenhouse condition with 70–80 % RH and 26 ± 2 °C temperature by removing the plastic bags. Finally, the plantlets were moved to greenhouse condition with 60–70 % RH and 28 ± 3 °C temperature and were kept for two more weeks. The plantlets were misted and irrigated frequently. They were also sprayed with 1/8 (in the first week) to 1/4 MS solution (in the second week) of primary acclimatization as source of energy until they start photosynthesis. Plantlets survived primary acclimatization (n = 325) were transferred to nursery shade-house and direct sunlight for three weeks for secondary acclimatization. The plantlets were watered twice a day. In all cases, survival and establishment rates were recorded.

### 2.5 Data analyses

Required data were collected from all experiments. All *in vitro* treatments were carried out in triplicates. Quantitative data were analyzed using relevant descriptive and inferential statistical methods using SPSS Version 20 software. Inferential (sample) data were analyzed using the analysis of variance (ANOVA) at *a priori* set *p-*value of ≤0.05. Post-hoc comparisons of means (±SD) were carried out using Least Significance Difference (LSD). Qualitative data collected by visual observations were used to strengthen results of quantitative data analyses.

## 3 Results and discussion

### 3.1 Initiation of *A. monticola* explants

This experiment was conducted to help the explants resume growth and other cellular activities and prepare them for the regeneration experiment. The resumption of such cellular activities was confirmed by the development of swelling at the bases of the explants. In some cases, explants can develop shoots due to their endogenous PGRs. The responses of *A. monticola* explants to different combinations and concentrations BAP and IBA supplements exhibited growth resumption and shooting.

Explants of the species were initiated in 9–29 days. Initiation media supplemented with 0.10 mg/LBAP resulted in initiation of explants in 9 days while the control (unsupplemented) resulted in initiation in 29 days (Table 1). Of the 22 initiation treatments, half of them resulted in explant initiation in less than 20 days. BAP is the most commonly used PGR for initiation of explants in aloes and other species [15,16,19]. The use of a wide range of concentrations (0.10−1.0 mg/L) of BAP alone or in combination with a constant concentration (0.10 mg/L) of NAA did neither show any difference nor pattern in affecting the mean days of initiation. This might be due to age-related variations in the explants because they cannot be of the same age [20]. The quicker initiation response in some treatments might be related to younger age of the explants rather than the PGR supplements.

**Table 1:** Initiation of *A. monticola* explants in different concentrations of BAP and IBA.

SN	PGRs (mg/L)		Mean (±SD) initiation responses		
	BAP	IBA	Days to initiation (*n* = 3)	No. of initiated explants (*n* = 3)	No. of shoots per explant (*n* = 3)
1	0.00	0.00	28.67 ± 0.58^a^	2.67 ± 0.58^a^	0.00 ± 0.00^c^
2	0.10	0.00	9.00 ± 0.00^m^	3.00 ± 0.00^a^	3.33 ± 0.58^a^
3	0.20	0.00	15.00 ± 1.73^i−k^	3.00 ± 0.00^a^	0.67 ± 0.58^bc^
4	0.30	0.00	21.00 ± 1.73^e^	2.67 ± 0.58^a^	0.33 ± 0.58^bc^
5	0.40	0.00	21.00 ± 1.00^e^	2.67 ± 0.58^a^	0.00 ± 0.00^c^
6	0.50	0.00	13.67 ± 0.58^kl^	2.67 ± 0.58^a^	0.67 ± 0.58^bc^
7	0.60	0.00	17.33 ± 2.52^f−h^	2.67 ± 0.58^a^	0.00 ± 0.00^c^
8	0.70	0.00	21.00 ± 1.00^e^	3.00 ± 0.00^a^	1.00 ± 0.00^b^
9	0.80	0.00	16.67 ± 0.58^g−i^	2.67 ± 0.58^a^	0.33 ± 0.58^bc^
10	0.90	0.00	24.67 ± 0.58^b^	3.00 ± 0.00^a^	0.33 ± 0.58^bc^
11	1.00	0.00	21.67 ± 1.53^de^	3.00 ± 0.00^a^	0.33 ± 0.58^bc^
12	0.00	0.10	22.67 ± 1.16^c−e^	2.67 ± 0.58^a^	0.67 ± 0.58^bc^
13	0.10	0.10	28.67 ± 0.58^a^	2.67 ± 0.58^a^	0.33 ± 0.58^bc^
14	0.20	0.10	15.67 ± 0.58^h−j^	2.67 ± 0.58^a^	0.33 ± 0.58^bc^
15	0.30	0.10	23.33 ± 1.16^b−d^	2.67 ± 0.58^a^	0.33 ± 0.58^bc^
16	0.40	0.10	18.33 ± 0.58^fg^	3.00 ± 0.00^a^	0.33 ± 0.58^bc^
17	0.50	0.10	15.33 ± 0.58^i−k^	3.00 ± 0.00^a^	0.33 ± 0.58^bc^
18	0.60	0.10	14.33 ± 0.58^j−l^	2.67 ± 0.58^a^	1.00 ± 0.00^b^
19	0.70	0.10	18.67 ± 0.58^f^	2.67 ± 0.58^a^	0.33 ± 0.58^bc^
20	0.80	0.10	24.33 ± 1.16^bc^	3.00 ± 0.00^a^	0.67 ± 0.58^bc^
21	0.90	0.10	21.67 ± 1.16^de^	2.67 ± 0.58^a^	0.33 ± 0.58^bc^
22	1.00	0.10	13.00 ± 0.00^l^	3.00 ± 0.00^a^	1.00 ± 0.00^b^

Means (±SD) in the same column with different letters are statistically significantly different at p ≤ 0.05.

Three × three explants were cultured for initiation in each of the 22 treatments. Whereas nine of the treatments resulted in 100 % (9 out of 9) initiation, 13 of them resulted 89 % (8 out of 9) initiation (Table 1) − yielding a cumulative rate of initiation of 93.40 %. We can see that the initiation capacity of the species is excellent but the differences in mean number of initiated explants have no pattern. For example 5 of the 9 treatments that resulted in 100 % initiation showed initiation response in less than 20 days while 4 of the 9 did in 20–29 days. Likewise, 5 of the 9 treatments that resulted in 100 % initiation were supplemented with BAP alone while 4 of the 9 were supplemented with BAB in combination with 0.10 mg/L NAA. Thus, the degree of initiation of the explants of *A. monticola* in terms of mean number of initiated explants during the initiation experiment might be affected by age-related internal factors, size of explants, and genotypes [20].

Initiation media are formulated to trigger the resumption of growth of the explants under *in vitro* conditions. But explants that exhibited resumption of growth quicker would produce shoots. In line with this observation, some studies in *Aloe* species have reported shooting during initiation experiments [15,19]. In the present study, 19 (86.4 %) of the 22 treatments have produced microshoots during the initiation experiment. Of the 19 treatments, 10 (52.6 %) produced shoots in less than 20 days while the 9 (47.4 %) produced the same in 20–29 days. However, there were no any pattern with the other variables of initiation response (i.e., length of time to initiation and degree of initiation) and the supplementation of PGRs (i.e., BAP alone or in combination with IBA). Despite the absence of any patterns, 93.4 % of *A. monticola* explants cultured in initiation media have survived and resumed growth in 9–29 days. Only 13 (6.6 %) explants were failed due to rotting. This performance can be increased by collecting young and viable explants and using better cleaning and sterilization procedures.

### 3.2 Regeneration response of *A. monticola* explants

All the treatments with different concentrations and combinations of BAP and IBA have resulted in shooting. Initiated explants of *A. monticola* have grown new shoots in 13–29 days (Table 2; Fig. 1A–F). Generally speaking, shorter days to shooting were observed in the treatments supplemented with 1.0–3.0 mg/L BAP in combination with 0.50 mg/L IBA. Mean days to shooting in treatments supplemented with 1.00, 1.50, and 2.00 mg/L BAP in combination with 0.50 IBA were statistically significantly shorter than the rest of the treatments (*p* ≤ 0.05). Several authors have reported shooting responses of various *Aloe* spp. in two weeks with BAP alone (a cytokinin) or in combination with other plant growth regulators such as IAA, IBA, and NAA (auxins) [15,16,19,[21], [22], [23], [24]].

**Table 2:** Shooting of *A. monticola* explants in full-strength MS media supplemented with BAP and IBA.

PGRs (mg/L)		Mean (±) shooting responses			
BAP	IBA	No. of days to shooting (*n* = 3)	No. of shoots per explant (*n* = 3)	Shoot length (cm) (*n* = 3).	No. of leaves per shoot (*n* = 3)
0.00	0.00	28.00 ± 1.00^a^	1.00 ± 0.00^f^	3.00 ± 0.00^f^	4.33 ± 0.57^c−e^
0.50	0.00	25.67 ± 0.57^bc^	2.00 ± 0.00^e^	3.33 ± 0.57^ef^	4.00 ± 0.00^d−f^
1.00	0.00	27.67 ± 1.15^ab^	2.00 ± 0.00^e^	3.33 ± 0.57^ef^	4.33 ± 0.57^c−e^
1.50	0.00	25.67 ± 2.08^bc^	2.00 ± 0.00^e^	4.33 ± 0.57^cd^	4.67 ± 0.57^b−d^
2.00	0.00	22.33 ± 0.57^de^	2.67 ± 0.57^d^	4.67 ± 0.57^cd^	5.00 ± 1.00^b−d^
2.50	0.00	24.67 ± 1.52^c^	2.00 ± 0.00^e^	4.00 ± 0.00^de^	4.33 ± 0.57^c−e^
3.00	0.00	20.00 ± 2.64^f^	3.00 ± 0.00^d^	5.00 ± 0.00^c^	5.33 ± 0.57^bc^
0.00	0.50	29.00 ± 1.00^a^	2.00 ± 0.00^e^	9.33 ± 0.57^a^	4.67 ± 0.57^b−d^
0.50	0.50	29.33 ± 1.15^a^	1.00 ± 0.00^f^	2.00 ± 0.00^g^	3.33 ± 0.57^e−g^
1.00	0.50	14.00 ± 0.00^g^	4.00 ± 0.00^c^	4.33 ± 0.57^cd^	5.67 ± 1.15^b^
1.50	0.50	13.67 ± 0.57^g^	5.00 ± 0.00^b^	4.00 ± 0.00^de^	5.33 ± 0.57^bc^
2.00	0.50	13.33 ± 0.57^g^	7.00 ± 0.00^a^	3.00 ± 0.00^f^	9.00 ± 0.00^a^
2.50	0.50	19.67 ± 0.57^f^	3.67 ± 0.57^c^	7.00 ± 1.00^b^	3.00 ± 0.00^fg^
3.00	0.50	21.00 ± 0.00^ef^	4.00 ± 0.00^c^	6.33 ± 0.57^b^	2.67 ± 0.57^g^

Means (±SD) in the same column with different letters are statistically significantly different at p ≤ 0.05.

**Fig. 1:** Shooting responses of *A. monticola* explants under different treatments. **A**: Control, **B**: 1.00 mg/L BAP, **C**: 2.00 mg/L BAP +0.50 mg/L IBA, **D**: 2.00 mg/L BAP; **E**: 3.00 mg/L BAP, **F**: 3.00 mg/L BAP +0.50 mg/L IBA.

Of the 14 regeneration treatments, 12 (86 %) of them have produced at least two shoots per explant. Five treatments supplemented with 1.00–3.00 mg/L BAP and 0.50 mg/L IBA have produced 3.67 (±0.57) to 7.00 (±0.00) shoots per explant. The mean shoot numbers of these treatments were statistically significantly greater than the rest of the nine treatments (Table 2; *p* ≤ 0.05). The control and the treatment supplemented with 0.50 mg/L BAP and 0.50 mg/L IBA produced the smallest mean number of shoot per explant (i.e., one shoot per explant). The use of various combinations of cytokinin and auxin supplements is a usual approach in formulating tissue culture media for better regeneration responses. Thus, MS media supplemented with combination of BAP and various auxins such as IAA, IBA, and NAA have yielded better shooting responses in many *Aloe* species [19,22,[25], [26], [27], [28], [29], [30], [31], [32]].

Shoot length and leaf number can be considered as good variables for estimating biomass in a given *Aloe* species [33]. Thus, explants with longer normal shoots and/or more leaves have more biomass. The mean shoot lengths of all regeneration treatments ranged from 2.00 (±0.00) to 9.33 (±0.57) cm. On the other hand, treatments supplemented with 1.00–3.00 mg/L BAP and 0.50 mg/L IBA yielded mean shoot lengths of 3.00 (±0.00) to 7.00 (±1.00) cm. Since the IBA-supplemented treatments have more shoots than the IBA-unsupplemented treatments, their total shoot lengths are greater than that of the IBA-unsupplemented ones. Likewise, the mean numbers of leaves per shoot of the treatments ranged from 2.67 (±0.57) to 9.00 (±0.00). Three of the five treatments with mean leaf number of 5.00 or more were the treatments supplemented with 1.00, 1.50, and 2.00 mg/L BAP in combination with 0.50 mg/L IBA. Owing to higher number of shoots, the total number of leaves in these treatments ranged from few to several dozen (Table 2). Hence, propagation media supplemented with 1.00–3.00 mg/L BAP in combination with 0.50 mg/L IBA were better in causing quick and profound regeneration in *A. monticola* in agreement with findings of many other studies [15,16,19,21].

### 3.3 Rooting response of *A. monticola* shoots

All the treatments have resulted in the rooting of the microshoots and yielded plantlets. Shoots or microshoots of *A. monticola* have yielded roots in 16–29 days (Table 3; Fig. 2A–F). Despite the pattern lacks consistency, the mean days to rooting of the shoots decreased with increasing the concentration of NAA supplements from 0.25 to 4.00 mg/L when applied alone or in combination with 0.25 mg/L IBA. Many studies have reported that NAA and other auxins are excellent PGRs in causing quick and extensive rooting in aloes [15,16,19,21,25,31,34]. Shorter mean days to rooting were observed in the treatments supplemented with 0.25 mg/L IBA. Half of the treatments supplemented with NAA in combination with 0.25 mg/L IBA yielded rooting in less than 20 days. Studies on *A. barbadensis* and *A. vera* reported quicker rooting response when NAA and IBA were applied in combination [26,35].

**Table 3:** Rooting of *A. monticola* shoots in half-strength MS media supplemented with NAA and IBA.

PGRs (mg/L)		Mean (±) rooting responses			
NAA	IBA	Number of days to rooting (*n* = 3)	Number of roots per shoot (*n* = 3)	Root length (cm) (*n* = 3)	Number of leaves per plantlet (*n* = 3)
0.00	0.00	29.00 ± 1.00^ab^	1.89 ± 0.19^ij^	1.10 ± 0.20^g^	3.11 ± 0.38^e−g^
0.50	0.00	28.00 ± 0.00^b^	5.56 ± 0.38^h^	2.61 ± 0.24^f^	3.33 ± 1.00^d−g^
1.00	0.00	24.33 ± 0.58^cd^	6.89 ± 0.51^g^	3.09 ± 0.14^ef^	2.33 ± 0.58^g^
1.50	0.00	24.67 ± 0.58^c^	9.11 ± 0.84^f^	3.33 ± 0.04^a^	4.00 ± 1.00^c−f^
2.00	0.00	23.33 ± 0.58^de^	9.89 ± 0.19e^f^	3.97 ± 0.25^d^	4.00 ± 0.00^c−f^
2.50	0.00	21.67 ± 0.58^f^	10.56 ± 0.77^e^	4.69 ± 0.53^c^	3.00 ± 1.00^fg^
3.00	0.00	23.00 ± 0.00^e^	10.44 ± 0.51^e^	6.44 ± 0.50^a^	4.33 ± 0.58^cd^
3.50	0.00	21.33 ± 0.58^f^	11.89 ± 0.51^d^	5.68 ± 0.19^b^	4.00 ± 0.00^c−f^
4.00	0.00	23.33 ± 1.15^de^	12.11 ± 0.77^d^	5.10 ± 0.26^c^	3.00 ± 0.00^fg^
0.00	0.25	29.33 ± 0.58^a^	1.33 ± 0.58^j^	0.32 ± 0.19^h^	3.33 ± 0.58^d−g^
0.50	0.25	28.00 ± 0.00^b^	2.67 ± 0.58^i^	1.57 ± 0.37^g^	4.00 ± 0.00^c−f^
1.00	0.25	15.67 ± 0.58^h^	14.67 ± 0.58^a^	5.89 ± 0.16^b^	7.67 ± 0.58^a^
1.50	0.25	21.00 ± 1.00^f^	12.67 ± 0.67^cd^	3.22 ± 0.46^e^	3.67 ± 0.58^d−f^
2.00	0.25	18.33 ± 0.58^g^	13.44 ± 0.19^bc^	3.96 ± 0.04^d^	6.67 ± 0.58^b^
2.50	0.25	23.67 ± 0.58^c−e^	9.89 ± 0.51^ef^	4.56 ± 0.30^c^	6.00 ± 0.00^b^
3.00	0.25	21.33 ± 0.58^f^	12.00 ± 0.00^d^	3.51 ± 0.17^de^	3.67 ± 0.58^d−f^
3.50	0.25	16.00 ± 0.00^h^	12.67 ± 0.58^cd^	4.83 ± 0.51^c^	5.00 ± 0.00^c^
4.00	0.25	18.56 ± 0.77^g^	14.33 ± 0.58^ab^	3.91 ± 0.27^d^	4.11 ± 0.19^c−e^

Means (±SD) in the same column with different letters are statistically significantly different at p ≤ 0.05.

**Fig. 2:** Rooting response of *A. monticola* shoots under different treatments. **A**: 4.00 mg/L NAA, **B**: 3.00 mg/L NAA and 0.25 mg/L IBA, **C**: 2.00 mg/L NAA +0.25 mg/L IBA, **D**: 1.00 mg/L NAA and 0.25 mg/L IBA; **E**: 4.00 mg/L NAA and 0.25 mg/L IBA, **F**: 1.00 mg/L NAA +0.25 mg/L IBA.

Among the treatments supplemented with NAA only, mean root number per shoot increased from 5.56 (±0.38) to 12.11 (±0.77) with increasing the NAA supplement from 0.50 to 4.00 mg/L (Table 3; Fig. 2A–F). The mean root length also showed steady increments with increasing NAA supplementation. This implies that increasing NAA supplementation from 0.50 to 4.00 mg/L enhances rooting of *A. monticola* through producing more and long roots (i.e., more biomass). On the other hand, treatments supplemented with 1.00–4.00 mg/L NAA in combination with 0.25 mg/L IBA yielded 9.89 (±0.51) to 14.67 (±0.58). Even though the total root biomass is still high, no clear increment was observed in terms of mean root length among these IBA supplemented treatments. This observation shows that the supplementation of IBA promotes the effects of NAA and enhances the rooting response of the species as observed in other studies [26,35].

Well-rooted shoots developed into plantlets that can be subjected to *ex vitro* acclimatization tests. The treatments supplemented with NAA alone produced plantlets with 2.33 (±0.58) to 4.33 (±0.58) mean leaves per plantlet. Though the pattern was not consistent, increasing the concentration of NAA led to increased mean leaf number per plantlet. On the other hand, treatments supplemented with 0.50–4.00 mg/L NAA in combination with 0.25 mg/L produced plantlets with mean leaf number of 3.67 (±0.58) to 7.67 (±0.58) per plantlet. This observation is a good indication that IBA supplementations to NAA treatments resulted in increased root biomass that led to enhanced leaf formation (shoot biomass).

### 3.4 Acclimatization response of *A. monticola* plantlets

Four weeks of primary acclimatization in coco peat produced 325 (ca. 98 %) survived and hardened plantlets (Table 4, Fig. 3A–F). Qualitative study via visual inspection of the six failed plantlets showed that the cause of their deaths was rotting. Comparably high rates of survival to primary acclimatization were reported in many species of *Aloe* including *A. trichosantha*, *A. elegans*, *A. adigratana*, *A. percrassa*, *A. vera*, and *A. barbadenesis* [15,16,19,21,22,36,37]. The high survival rate in primary acclimatization may be accounted to the coco peat planting material. Its spongy-like characteristics with high water and air holding capacity can help the plantlets to produce good root system quickly [19].

**Table 4:** *Ex vitro* acclimatization performance of *A. monticola* plantlets.

Acclimatization condition			Acclimatization responses		
Type	Planting material^a^	Lighting conditions	Planted plantlets (*n*)	Established plantlets	
				Quantity (*n*)	Percent
Primary	Cocopeat	Greenhouse	331	325	98
Secondary	Composted soil	Nursery shade	80	73	91
		Direct sunlight	78	70	90
	Manured soil	Nursery shade	84	80	95
		Direct sunlight	83	78	94

a Composted soil: Soil, sand, and compost at 1:1:1 ratio; Manured soil: Soil, sand, and manure at 1:1:1 ratio.

**Fig. 3:** *Ex vitro* acclimatization of performance *A. monticola* plantlets under different planting materials and lighting conditions **A.** Plantlets obtained from control; **B**. Plantlets obtained from 1 mg/L NAA and 0.25 mg/LIBA; **C**. Plantlets after 10 days of greenhouse acclimatization; **D.** Plantlets after 21 days of greenhouse acclimatization; **E**. Plantlets in manured soil; **F.** Plantlets in composted soil.

Secondary acclimatization experiments are carried out by modifying the planting materials, the lighting conditions, and/or both. Secondary acclimatization of *A. monticola* in composted and manured planting materials under nursery shade and direct sunlight showed 90–95 % survival rates after three weeks (Table 4). However, secondary acclimatization with manured soil as planting material produced slightly better results than with composted soil (Table 4). The effect of lighting was very small with 1 % difference in survival. *Ex vitro* acclimatization of *Aloe* plants often yields high rate of success as reported in many studies [19,22,23,25,29,31,[37], [38]].

## 4 Concluding remarks

*A. monticola* is restricted to some mountain peaks of Ethiopia's Tigrai floristic region. Limited stands are available in some pockets in Aiba and Giorgis Belonta, North of Maichew city. Like the other species, *A. monticola* is planted as life fences of backyards, farmlands, churchyards, footpaths, mountain terraces, and area enclosures as well as demarcations of farmlands. Field observation in the aforementioned locations showed that this ecologically and environmentally restricted and endangered plant has very limited natural regeneration capacity. Offshoots and young plants were not common. Young plants were partly eaten by grazing animals and livestock. Thus, the present study has provided excellent insights into artificial propagation of the plant. The findings are important for developing refined protocol of *in vitro* micropropagation of *A. monticola* by focusing on establishing the best combination of NAA and IBA supplementation. The protocol will be an important tool for mass propagation of the plant to rehabilitate mountainous and alpine habitats in northeastern Ethiopia. Such an endeavor can contribute to local and national programs of conservation of biological and genetic diversity.

## Data availability statement

The data will be made available on request.

## CRediT authorship contribution statement

**Birhanu Debesay Berhe:** Conceptualization, Data curation, Formal analysis, Investigation, Methodology, Software, Writing – original draft. **Desta Berhe Sbhatu:** Conceptualization, Data curation, Funding acquisition, Methodology, Project administration, Resources, Supervision, Validation, Writing – review & editing. **T. Mohammad Munawar:** Conceptualization, Methodology, Resources, Software, Validation. **Gebreselama Gebreyohannes:** Conceptualization, Methodology, Resources, Software, Visualization.

## Declaration of competing interest

The authors declare that they have no known competing financial interests or personal relationships that could have appeared to influence the work reported in this paper.
